# PredAmyl-MLP: Prediction of Amyloid Proteins Using Multilayer Perceptron

**DOI:** 10.1155/2020/8845133

**Published:** 2020-11-20

**Authors:** Yanjuan Li, Zitong Zhang, Zhixia Teng, Xiaoyan Liu

**Affiliations:** ^1^College of Information and Computer Engineering, Northeast Forestry University, Harbin 150040, China; ^2^College of Computer Science and Technology, Harbin Institute of Technology, Harbin 150040, China

## Abstract

Amyloid is generally an aggregate of insoluble fibrin; its abnormal deposition is the pathogenic mechanism of various diseases, such as Alzheimer's disease and type II diabetes. Therefore, accurately identifying amyloid is necessary to understand its role in pathology. We proposed a machine learning-based prediction model called PredAmyl-MLP, which consists of the following three steps: feature extraction, feature selection, and classification. In the step of feature extraction, seven feature extraction algorithms and different combinations of them are investigated, and the combination of SVMProt-188D and tripeptide composition (TPC) is selected according to the experimental results. In the step of feature selection, maximum relevant maximum distance (MRMD) and binomial distribution (BD) are, respectively, used to remove the redundant or noise features, and the appropriate features are selected according to the experimental results. In the step of classification, we employed multilayer perceptron (MLP) to train the prediction model. The 10-fold cross-validation results show that the overall accuracy of PredAmyl-MLP reached 91.59%, and the performance was better than the existing methods.

## 1. Introduction

Amyloid is an insoluble fibrous protein formed by the aggregation of certain misfolded proteins [1]. They are found in bacteria, fungi, yeast, and mammals [2]; the diversity of functions is comparable to soluble proteins. Amyloid proteins play an important role in the formation of biofilms [3], the binding and storage of peptide hormones [4], antimicrobial activity [5], and the antiviral innate immune response [6]. But not all amyloid proteins are beneficial, the extracellular deposition of amyloid fibrils can cause a series of diseases such as Alzheimer's diseases [7], type II diabetes, and Parkinson's disease [8, 9]. To understand amyloid proteins and related diseases deeply, researchers have carried out a lot of work on amyloid proteins, including amyloidosis [10, 11], polymorphs of amyloid proteins at the molecular level [12], amyloid region [13], and antibody amyloid [14].

Studies have shown that not all regions of polypeptides contribute equally to its aggregation; only some short specific amino acid sequences can act as facilitators of amyloid fibril formation [15, 16]. Therefore, many computational methods for detecting the amyloid-forming regions have been proposed. AGGRESCAN [17] is a web tool, which identifies the aggregation-prone regions in the sequence based on the intrinsic aggregation-prone profile of amino acids and their relative positions. Due to its dependence on the analysis of linear sequences, it is difficult for AGGRESCAN to predict the aggregation properties of folded proteins. Zambrano et al. improve AGGRESCAN and propose a new method called AGGRESCAN3D (A3D for short) [18]. By using many factors affecting protein aggregation, A3D obtains a more accurate prediction for globular proteins. Zyggregator [19] predicts the aggregation-prone regions of polypeptides based on the physical and chemical properties of protein primary structure, such as hydrophobicity and secondary structure tendency. Based on the formation mechanism of *β*-sheets in amyloid aggregates, PASTA [20] uses the energy function to calculate the amino acid fragments in the sequence. FoldAmyloid [21] introduces the expected probability of hydrogen bonds and the packing density of residues to detect the amyloidogenic regions in polypeptide chains. Maurer-Stroh's method [22] is a prediction algorithm using position-specific scoring matrices to determine amyloid formation sequences.

The prediction principles of the above methods are different and have their own advantages and disadvantages. The idea of combining different predictors to improve the identification ability was first introduced in AmylPred [23], subsequently followed by the improved version AmylPred2 [24]. AmylPred2 combines 11 different individual predictors to form a consensus prediction of the amyloidogenic region. The consensus of AmylPred2 is based on binary predictions; Emily et al. improves the weighting process and proposes MetAmyl [25]. MetAmyl introduces the meta-prediction whose input is the prediction scores of base-prediction based on a statistical approach.

In recent years, machine learning has increasingly become a favorite tool in the field of bioinformatics [26–35]. Many scholars try to use machine learning algorithms to predict amyloidogenic propensity. PASTA 2.0 [36] not only uses a pairwise energy potential to predict amyloid fibril regions but also uses machine learning algorithms to detect secondary structure. FISH Amyloid [37] proposes an original machine learning classification method to investigate co-occurrence patterns in the sequence based on the assumption that the distribution of residues in amyloid-forming fragments is position-specific. APPNN [38] is a phenomenological amyloid formation propensity predictor established on recursive feature selection and feed-forward neural network. Experimental results show that APPNN has a high accuracy value compared with other amyloidogenic propensity prediction methods.

These methods can help us understand amyloid-related diseases and find potential therapeutic targets. However, their work focuses on predicting the amyloid-forming region of a given sequence, rather than identifying whether this sequence is amyloid. Niu et al. propose RFAmyloid [39] to identify amyloid based on random forest, which obtains an accuracy of 89%. Although high accuracy has been achieved, there are still many aspects worthy of further investigation, such as redundant features due to no feature selection. In this paper, we aim to propose a new amyloid predictor, PredAmyl-MLP, to further improve the prediction performance.

## 2. Materials and Methods

### 2.1. Framework of PredAmyl-MLP

In this paper, we proposed a new amyloid predictor called PredAmyl-MLP, the framework of which is shown in Figure 1. First, we, respectively, extracted 188-dimensional vectors and 8000-dimensional vectors to represent protein sequences by using the SVMProt-188D method and the TPC method. Next, we reduced the 188-dimensional vectors to 121-dimensional vectors using the MRMD method, reduced 8000-dimensional vectors to 425-dimensional vectors using the BD method, and then generated multi-feature vectors by combining the 121-dimensional and 425-dimensional vectors. Finally, we constructed a multilayer perceptron-based classifier that takes the multi-feature vectors as input. We will introduce the datasets, feature extraction, feature selection, and classifiers in detail in the following section.

### 2.2. Dataset

In this study, we utilized the dataset constructed by Niu et al. who developed a web server named RFAmyloid [39] to identify amyloid proteins. There are three reasons for considering this dataset as our experimental dataset. First, the dataset was collected from the UniProt database (http://www.uniprot.org/) and the AmyPro database (http://www.amypro.net/); thus, it is reliable. Second, the authors employed the program CD-HIT [40] to cluster proteins that meet a similarity threshold and removed redundant and homology-biased sequences [41]. Finally, and most importantly, using the same dataset allows us to compare the proposed method fairly with existing methods. The final dataset consists of 165 amyloid proteins (positive examples) and 382 non-amyloid proteins (negative examples).

### 2.3. Feature Extraction

The first and the most important step of designing a protein predictor is how to represent protein by features that can effectively discriminate positive samples from negative samples [42–48]. In this paper, we try to encode amyloid proteins with multi-feature, which consists of two basic feature representation methods, namely, SVMProt-188D and Tripeptide compositions (TPC). SVMProt-188D is based on the composition and physicochemical properties of amino acids. It has achieved good performance on several bioinformatics applications such as human protein subcellular localization prediction [49–52], TATA binding protein identification [53], and protein functional family prediction [54–59]. TPC is based on the tripeptide composition of protein. It also has been widely applied to solve many bioinformatics problems such as hormone binding protein identification [60], the prediction of subcellular localization of mycobacterial proteins, and the identification of cancerlectins [61–63]. In this paper, we, respectively, extract SVMProt-188D and TPC features from a protein and combine the features to represent the protein. The experimental results show that the multi-feature can effectively encode the protein, which is shown in Section 3.2. The detail of SVMProt-188D and TPC is as follows.

#### 2.3.1. SVMProt-188D

Based on the composition and physicochemical properties of amino acids, the SVMProt-188D method encodes a protein as a 188-dimensional feature vector. The first 20 dimensions are represented by calculating the frequencies of 20 natural amino acids (A,C,D,E,F,G,H,I,K,L,M,N,P,Q,R,S,T,V,W,Y in alphabetical order) in the sequence. The formula can be defined as

(1) $$\begin{array}{c} \left(V_{1},V_{2},\cdots ,V_{20}\right)=\frac{N_{i}}{L}, \end{array}$$

where *N*_*i*_ represents the number of the *ith* amino acid in the protein sequence and *L* represents the length of a sequence. Obviously, ∑*V*_*i*_ = 1.

The latter dimensions are correlated with eight physicochemical properties including hydrophobicity, normalized Van der Waals volume, polarity, polarizability, charge, surface tension, secondary structure, and solvent accessibility. Each property is divided into three categories, and 20 amino acids belong to different categories (listed in Table 1). All physicochemical properties are described by three descriptors *C* (composition), *T* (transition), and *D* (distribution). The *C*, *T*, and *D* descriptors of each property consist of 3, 3, and 15 numbers, respectively. *C* is the frequency of amino acids in a specific category. *T* is the percent frequency that amino acids in a category followed by amino acids in another category, such as the transitions from hydrophilic to hydrophobic or from neutral to hydrophilic. *D* calculates the proportions of the chain length of the first, 25, 50, 75, and 100% amino acids in a specific category and enlarges the calculations by 100 times.

Therefore, after analyzing the composition and eight physicochemical properties of amino acids, we can obtain a total of 20 + (C + T + D) × 8 = 188 features.

#### 2.3.2. TPC

The TPC method represents sequences based on the tripeptide composition of protein. Three amino acids are linked by peptide bonds to form a tripeptide, thus producing 20 × 20 × 20 = 8000 possible tripeptides. TPC transforms 8000 tripeptides into an 8000-dimensional feature vector that can express a protein sequence. The formula is defined as follows:

(2) $$\begin{array}{c} F={\left[f_{1},f_{2},\cdots ,f_{8000}\right]}^{T}, \end{array}$$

where *T* is the transposition of a vector and *f*_*i*_ is the frequency of the tripeptide in the sequence, which can be calculated as

(3) $$\begin{array}{c} f_{i}=\frac{N_{i}}{L-2}, \end{array}$$

where *N*_*i*_ is the number of the *ith* tripeptide and *L* represents the length of a sequence.

### 2.4. Feature Selection

Feature selection plays an important role in the improvement of identification performance. It can remove redundant or noise features. We adopted the maximum relevant maximum distance (MRMD) [64] method to select optimal features from SVMProt-188D features and adopted the binomial distribution (BD) [65] method to select optimal features from TPC features. The principles of the two feature selection methods are as follows.

#### 2.4.1. MRMD

Most dimensionality reduction methods focus on the correlation between features and target class, ignoring the redundancy of features [64]. However, the effect of highly correlated feature vectors on classification cannot be superposed. The MRMD method considers these two aspects to score features. Therefore, the score for each feature contains two components, the maximum relevant MR score and the maximum distance MD score, which can be defined as

(4) $$\begin{array}{c} \max\left({\text{MR}}_{i}+{\text{MD}}_{i}\right). \end{array}$$

The relevance between feature and target class is measured by the Pearson correlation coefficient (PCC). The formula is defined as

(5) $$\begin{array}{c} PCC\left(\vec{F_{\text{i}}},\vec{C}\right)=\frac{\sum_{k=1}^{N}\left(F_{ik}-\bar{F_{i}}\right)\left(C_{k}-\bar{C}\right)}{\sqrt{\sum_{k=1}^{N}{\left(F_{ik}-\bar{F_{i}}\right)}^{2}}\sqrt{\sum_{k=1}^{N}{\left(C_{k}-\bar{C}\right)}^{2}}}, \end{array}$$

where *N* is total number of samples,$\vec{F_{i}}$ and $\vec{C}$ consist of the *ith* dimension feature vector and the corresponding target class *c* in each sample, respectively; *F*_*ik*_ and *C*_*k*_ is the *kth* element of $\vec{F_{i}}$ and $\vec{C}$, respectively. If this feature contributes significantly to classification, the value of |PCC| will be large. Thus, the MR score for feature *i* is calculated as

(6) $$\begin{array}{c} \max{\text{MR}}_{i}=\left|\text{PCC}\left(\vec{F_{i}},\vec{C}\right)\right|. \end{array}$$

The correlation between features is evaluated by calculating the distance between features. In this work, Euclidean distance (ED), Cosine similarity (COS), and Tanimoto coefficient (TC) are employed as distance functions. The formulas are as follows:

(7) $$\begin{array}{c} {\text{ED}}_{i}=\frac{\sum \sqrt{\sum_{k=1}^{M}{\left(F_{i}-F_{k}\right)}^{2}}}{M-1}\left(i\leq k\leq M,k\neq i\right),\\ {\text{COS}}_{i}=\frac{\sum F_{i}*F_{k}}{\left\|F_{i}\right\|*\left\|F_{k}\right\|*\left(M-1\right)}\left(i\leq k\leq M,k\neq i\right),\\ {\text{TC}}_{i}=\frac{\sum F_{i}*F_{k}}{\left({\left\|F_{i}\right\|}^{2}+{\left\|F_{k}\right\|}^{2}-F_{i}*F_{k}\right)*\left(M-1\right)}\left(i\leq k\leq M,k\neq i\right), \end{array}$$

and the MD score for feature *i* is defined as

(8) $$\begin{array}{c} \max{\text{MD}}_{i}=\frac{1}{3}\left({\text{ED}}_{i}+{\text{COS}}_{i}+{\text{TC}}_{i}\right). \end{array}$$

#### 2.4.2. BD

In this work, the binomial distribution method [66–68] was applied to select the optimal subset from 8000 tripeptide features. First, we judged whether the occurrence of tripeptides in a certain kind of protein is random by calculating the probability of the *ith* tripeptide in the class *j* samples, like this:

(9) $$\begin{array}{c} P_{ij}=\overset{N_{i}}{\underset{k=n_{ij}}{\sum }}\frac{N_{i}!}{k!\left(N_{i}-k\right)!}{q_{j}}^{k}{\left(1-q_{j}\right)}^{N_{i}-k}, \end{array}$$

where *q*_*i*_ is the proportion of the number of tripeptides in class *j* samples to in all samples, *n*_*ij*_ and *N*_*i*_ are the occurrence number of the *ith* tripeptide in class *j* (*j* = {0, 1}) and all samples, respectively. A smaller *P* value indicates more certainty about the occurrence of tripeptides. Hence, the confidence level (CL) of the *ith* tripeptide in the class *j* samples can be defined as

(10) $$\begin{array}{c} {\text{CL}}_{ij}=1-P_{ij}. \end{array}$$

Obviously, each tripeptide feature has two CL values, and we will choose the larger one.

Then, the features are arranged in descending order by CL values to create a ranked list. The first feature subset contains only the first feature in the list,*D*_1_ = [*f*_1_]^*T*^. And each new subset was produced when the next candidate feature was added to the previous subset. This process was repeated until all features in the list were added. The resulting 8000 feature subsets can be described as

(11) $$\begin{array}{c} D={\left[D_{1},D_{2},\cdots ,D_{8000}\right]}^{T}. \end{array}$$

Finally, for every feature set, a prediction model was constructed. The optimal feature subset can be selected based on the maximum accuracy of 10-fold cross-validation.

### 2.5. Classifier

Waikato Environment for Knowledge Analysis (Weka) is a well-known machine learning and data mining software. In the platform of Weka, we can integrate our own algorithms and even use his own algorithms to implement the classification task. In this paper, we experimented with many classification algorithms based on the Weka platform, such as random forest, naive Bayes, logistic, IBK, and bagging [69, 70]. Finally, we choose the multilayer perceptron (MLP) as our classifier, and the experimental results are shown in Section 3.3.

Artificial neural network is a machine learning algorithm that simulates the human brain. Multilayer perceptron is a kind of feedforward artificial neural network, which has a strong learning ability and robustness [71]. It performs very well in solving various practical problems and has been widely used in the field of bioinformatics, such as disease diagnosis [72, 73], the prediction of protein secondary structure [74], and gene classification [75]. MLP utilizes feature vectors as nodes in the input layer. In the training process, the output values are compared with the actual values, and error information is fed back. Based on the information, the weights continuously update until the prediction error is sufficiently small.  Figure 2 is a schematic diagram of MLP. In this work, we constructed an MLP model with one hidden layer. The number of neurons in the hidden layer is set to half of the sum of the number of input features and output classes. Meanwhile, the learning rate and the number of iterations are set to 0.3 and 500, respectively.

### 2.6. Measurement

To evaluate the performance of our prediction model, we used four indicators commonly used in bioinformatics: accuracy (ACC), sensitivity (SE), specificity (SP), and Mathew's correlation coefficient (MCC) [76–87]. These measures are formulated as follows:

(12) $$\begin{array}{c} \text{ACC}=\frac{\text{TP}+\text{TN}}{\text{TP}+\text{TN}+\text{FP}+\text{FN}},\\ \text{SE}=\frac{\text{TP}}{\text{TP}+\text{FN}},\\ \text{SP}=\frac{\text{TN}}{\text{TN}+\text{FP}},\\ \text{MCC}=\frac{\text{TP}\times \text{TN}‐\text{FP}\times \text{FN}}{\sqrt{\left(\text{TP}+\text{FP}\right)\left(\text{TP}+\text{FN}\right)\left(\text{TN}+\text{FP}\right)\left(\text{TN}+\text{FN}\right)}}, \end{array}$$

where TP is the abbreviation of true positive, which means the number of amyloid proteins predicted in the positive samples; FP is the abbreviation of false positive, which means the number of amyloid proteins predicted in the negative samples; TN is the abbreviation of true negative, which means the number of non-amyloid proteins predicted in the negative samples; and FN is the abbreviation of false negative, which means the number of non-amyloid proteins predicted in the positive samples. The SE and SP, respectively, denote the predictive ability of a model in positive and negative samples. Both ACC and MCC denote the overall performance of a model. For all the indicators mentioned above, the higher scores they achieve, the better performance the models have.

## 3. Results and Discussion

### 3.1. Experiments on Feature Selection

As described in Framework of PredAmyl-MLP, we, respectively, extract SVMProt-188D and TPC features from samples and encode each sample with a multi-feature of 8188 dimensions. Training a classification model using too many feature vectors with low confidence will be relatively time-consuming, and the model may be overfitting. On the contrary, if the number of feature vectors is too small, they will not afford enough information to discriminate positive samples from negative samples. Therefore, to construct a robust and efficient prediction model, we, respectively, adopt MRMD and BD methods to choose an appropriate number of features from SVMProt-188D and TPC features. In this section, we will give the process of feature selection and experimental results.

For the 188-dimensional features extracted by the SVMProt-188D method, we assessed their importance by calculating the MRMD scores. The feature with a higher score has a more significant contribution to amyloid identification. The MRMD score consists of the Pearson correlation coefficient and distance function. The MRMD method provides three distance functions including Euclidean distance (ED), Cosine similarity (COS), and Tanimoto coefficient (TC). Different distance functions will lead to different MRMD scores for each feature. Thus, choosing an appropriate distance function is crucial for removing redundant features.

We employed support vector machines (SVM) [88, 89], a powerful classification algorithm, to examine the performance of three distance functions and select an optimal feature subset. First, we ranked the features in decreasing order of the MRMD scores to obtain the feature list. Then, we built feature subsets according to the feature order in the list. The first set contains only the feature ranking first in the list. A new set was generated when the second feature was added to the previous set. This process was repeated until all candidate features were added. Finally, the constructed 188 subsets were input into an SVM-based classifier, and the 10-fold cross-validation accuracy was obtained.

Figure 3 illustrates the performance of MRMD based on different distance functions, where MEAN represents the average of three distance function. As shown in Figure 3, ED, COS, TC, and MEAN have the best predictive performance when using the top-ranked 121, 174, 177, and 121 features, respectively. Furthermore, the results obtained by ED distance function are almost identical to those obtained by the average of different distance functions. It suggests that the method using ED distance function can achieve the same effect as using the average of the three distance functions. Although the maximum accuracy of TC is slightly higher than that of ED, the number of features required for ED to obtain the best performance is much lower than that of TC. Therefore, we adopted ED as the distance function of the MRMD method and used the top 121 features in the ED ranking list to construct an optimal feature subset.

Figure 4 presents the MRMD score of each feature calculated using ED distance function, where the features marked with red are selected and the ones marked with blue are removed. As we can see from Figure 4, most of the redundant features appear continuously and concentratedly, such as 21-26, 42-47, 126-131, 147-152, and 168-175. We analyzed the reasons and found that these features were extracted based on the content of three categories of amino acids in the sequences and the transition frequency between every two categories. Such features are regarded as redundant features, possibly because they are insensitive to identifying amyloid or encodes very similar. This discovery also brings new ideas for our future research.

For the 8000 features extracted by the TPC method, we sorted them using the BD method. According to the sort order, a certain number of features are selected and formed a feature subset. Thus, we can construct 8000 feature subsets. For each subset, the SVM classifier trained with 10-fold cross-validation. The relationship between the accuracy and the number of features is shown in Figure 5. As shown in Figure 5, the accuracy reaches a maximum of 91.22% when the number of features is 1565. This number is much larger than the number of 547 samples in our dataset. The construction of a robust prediction model must take into account the time-consuming and risk of overfitting caused by high-dimensional feature vectors. Ultimately, we chose the top 425 features which can achieve an overall accuracy of 87.93% which was just slightly lower than the maximum accuracy (91.22%) produced by the top 1565 features. Therefore, the top 425 features served as the optimal feature subset in the TPC feature method.

In summary, we, respectively, selected 121 features from SVMProt-188D features and 425 features from TPC features, then combined the 121 features and 425 features to form a multi-feature which consists of 546 features. The multi-feature is used to train the multilayer perceptron classifier in this study.

### 3.2. Performance of Different Features

As shown in Experiments on Feature Selection, we, respectively, extracted 188-dimensional vectors and 8000-dimensional vectors from protein sequences by using the SVMProt-188D method and the TPC method. Next, we reduced the 188-dimensional vectors to 121-dimensional vectors using the MRMD method, reduced 8000-dimensional vectors to 425-dimensional vectors using the BD method, and then generated multi-feature vectors by combining the 121-dimensional and 425-dimensional vectors. We used the multi-feature with dimensions of 546 to represent samples.

To verify the validity of the multi-feature used in this paper, we first used multilayer perceptron as the classifier and compared the multi-feature with some other features, including *k*-skip-2-gram [90], pseudo amino acid composition (PseAAC) [91], conjoint triad (CTriad) [92], dipeptide composition (DPC) [93], and 473D [94]. Then, three compared features with higher accuracy were combined and evaluated. Both PseAAC and DPC are based on amino acid composition. PseAAC takes into account the local information and long-range correlation of sequences. DPC represents a protein sequence through dipeptide composition information. *N*-gram is a common model in natural language processing, and *k*-skip-*n*-gram integrates the distance information between *n* residues into the traditional *n*-gram model. CTriad is a feature extraction method based on the neighbor relationship of amino acids. 473D encodes a sequence into a 473-dimensional feature vector based on the PSI-BLAST [95] and PSI-PRED [96] profiles.

The 10-fold cross-validation results are shown in Table 2, where both SVMProt-188 and TPC denote the final feature after feature selection. As shown in Table 2, from the indicators of ACC and MCC, the combination of SVM-188D and TPC used in this paper performs better than all other methods and has a better overall performance. According to the indicator of SE, our multi-feature also has the highest value, which demonstrates that our method performs better than other methods in identifying amyloid proteins from positive samples. According to the indicator of SP, our method is slightly lower than TPC, 473D, and the combination of CTriad and 473D. However, the values of ACC, MCC, and SE of our method are obviously higher than theirs. Especially the SE of 473D and the combination of CTriad and 473D are 0.339 and 0.036, respectively, which verify that they are biased to classify proteins as non-amyloid protein. Therefore, from the overall perspective, our method obviously performs better than all other methods.

To further illustrate that our multi-feature method has better performance regardless of the classifier, we, respectively, compared our multi-feature method with other feature extraction methods based on six different classifiers. The result is shown in Figure 6. As we can see from Figure 6, in each group of models using the same classifier, the accuracy of the combination of SVMProt 188-D and TPC is significantly higher than other feature extraction methods. Taking the classifier SGD as an example, the accuracy of the combination of SVMProt 188-D and TPC is about 9-16% higher than other methods. In general, our multi-feature method has better performance regardless of the classifier.

### 3.3. Performance of Different Classifiers

The selection of a classification algorithm is an important step to improve the accuracy of the model. Based on the multi-feature used in this paper, we compared multilayer perceptron with ten popular classifiers, including random forest, naïve Bayes, decision tree, AdaBoostM1, logistic, SGD, LibSVM, IBK, LWL, and bagging. SGD is a linear classifier using a stochastic gradient descent optimization algorithm. Naïve Bayes is based on Bayes' theorem and assumes that the features are independent and equally important. LibSVM is a software developed by Lin et al. to implement SVM. Logistic establishes a regression equation for the decision boundary based on the training data and classifies the test data accordingly. Decision tree divides test datasets based on the concept of entropy in informatics. AdaBoost, bagging, and random forest are ensemble classifiers. AdaBoost is an adaptive iterative algorithm, which integrates multiple weak classifiers trained on the same dataset into a strong classifier. Bagging is a parallel ensemble learning method based on bootstrap sampling. It trains a base classifier for each sampled dataset and then combines the base classifiers. Random forest is an extended variant of bagging that uses decision trees as the base classifier and introduces random attribute selection. Both IBK and LWL are lazy learning algorithms, which mean that the model is trained after receiving a test sample. IBK works by finding the *k* training samples nearest to a given test sample and determine the category of the given sample based on these *k* “neighbors,” while LWL adds a concept of weighting. The results of 10-fold cross-validation are shown in Table 3.

In Table 3, although the multilayer perceptron method presented in this paper is slightly lower than IBK in the SP index, multilayer perceptron is obviously superior in the other three indices. In the indicator of SE, naïve Bayes achieved higher value than multilayer perceptron, but in the other three indicators of ACC, SP, and MCC, multilayer perceptron is superior to naïve Bayes. According to the indicators of ACC and MCC, multilayer perceptron is higher than all other classifiers. In general, the multilayer perceptron classifier used in this paper has better performance than other classifiers, which demonstrates that our method is effective in identifying amyloid.

### 3.4. Comparison with Other Methods

To further evaluate the performance of PredAmyl-MLP, we compared it with two state-of-the-art methods such as RFAmyloid [39] and BioSeq-Analysis [97] on the same dataset. BioSeq-Analysis is a platform of DNA, RNA, and protein sequence analysis that is available online at http://bioinformatics.hitsz.edu.cn/BioSeq-Analysis/PROTEIN. The SVM and random forest algorithm are used in the BioSeq-Analysis prediction method, we compared them separately. The comparison results are shown in Table 4. As we can see from Table 4, our predictor outperforms the other methods in all indicators. Furthermore, Figure 7 plots the ROC curves of the four methods. We can also see that PredAmyl-MLP is superior to existing methods in the prediction of amyloid.

## 4. Conclusions

In this paper, we proposed a novel model for identifying amyloid proteins, called PredAmyl-MLP. We used the SVMProt-188D and the Tripeptide composition methods to represent protein sequences, respectively. After removing redundant features, a multilayer perception-based prediction model was constructed using mixed feature vectors. To validate the performance of PredAmyl-MLP, we compared different feature subsets, classifiers, and other methods. As a result, the features after dimension reduction can achieve better performance. Moreover, the combination of two feature representation methods significantly improves accuracy. Through a lot of experiments, PredAmyl-MLP achieved an accuracy of 91.59%, and MCC reached 0.798, outperforming other existing methods. The online server for this article is available at http://106.12.83.135:8080/amyWeb_Release/index.jsp.

In future work, we will optimize the feature representation method, using lower-dimensional feature vectors to represent amyloid sequences. Moreover, we will consider other computational intelligence models [98–102] and optimization methods [103–105] for amyloid prediction.

## Figures and Tables

**Figure 1:** The frame chart of the PredAmyl-MLP predictor.

**Figure 2:** The structure of MLP with one hidden layer.

**Figure 3:** Comparison of different distance functions.

**Figure 4:** The MRMD scores of 188 features extracted by the SVMProt-188D method.

**Figure 5:** The accuracies of models built with different number of features.

**Figure 6:** The accuracy of various feature extraction methods using different classifiers.

**Figure 7:** ROC curve for PredAmyl-MLP and other methods.

**Table 1:** Three groups of amino acids divided by 8 different physicochemical properties.

Physicochemical property	Class1	Class2	Class3
Hydrophobicity	RKEDQN	GASTPHY	CVLIMFW
Normalized Van der Waals volume	GASCTPD	NVEQIL	MHKFRYW
Polarity	LIFWCMVY	PATGS	HQRKNED
Polarizability	GASDT	CPNVEQIL	KMHFRYW
Charge	KR	ANCQGHILMFPSTWYV	DE
Surface tension	ILMFPWYV	KTSEC	GQDNAHR
Secondary structure	EALMQKRH	VIYCWFT	GNPSD
Solvent accessibility	ALFCGIVM	RKQEND	MPSTHY

**Table 2:** Comparison of different feature representation methods.

Method	ACC (%)	SE	SP	MCC
SVMProt-188D+TPC	91.59	0.836	0.950	0.798
PseAAC+473D	64.71	0.339	0.780	0.126
PseAAC+CTriad	72.76	0.491	0.830	0.333
CTriad+473D	70.56	0.036	0.995	0.119
473D+PseAAC+CTriad	67.45	0.230	0.866	0.120
SVMProt-188D	80.80	0.606	0.895	0.527
TPC	90.12	0.776	0.955	0.760
*k*-skip-2-gram	71.11	0.291	0.893	0.228
PseAAC	78.42	0.570	0.877	0.469
CTriad	72.57	0.345	0.890	0.281
DPC	68.37	0.345	0.830	0.193
473D	76.96	0.339	0.955	0.398

**Table 3:** Comparison of multilayer perceptron with other classifiers.

Method	ACC (%)	SE	SP	MCC
Multilayer perceptron	91.59	0.836	0.950	0.798
Random forest	85.00	0.642	0.940	0.629
Naïve Bayes	86.28	0.848	0.869	0.692
Decision tree	79.52	0.618	0.872	0.503
AdaBoostM1	82.81	0.612	0.921	0.574
Logistic	87.93	0.721	0.948	0.705
SGD	89.57	0.776	0.948	0.747
LibSVM	74.95	0.424	0.890	0.357
IBK	79.52	0.376	0.976	0.481
LWL	81.35	0.594	0.908	0.537
Bagging	83.36	0.588	0.940	0.585

**Table 4:** Comparison of our method with other existing methods.

Method	ACC (%)	SE	SP	MCC
PredAmyl-MLP	91.59	0.836	0.950	0.798
RFAmyloid	89.19	0.781	0.927	0.739
BioSeq (RF)	81.31	0.6374	0.8989	0.5626
BioSeq (SVM)	76.86	0.4953	0.9006	0.4419

## Data Availability

The datasets used during the present study are available from the corresponding author upon reasonable request, or can be downloaded from http://106.12.83.135:8080/amyWeb_Release/index.jsp
